# Effect of Ultrasound-Guided Fascia Iliac Compartment Block on Serum NLRP3 and Inflammatory Factors in Patients with Femoral Intertrochanteric Fracture

**DOI:** 10.1155/2022/1944659

**Published:** 2022-05-17

**Authors:** Kailai Zhu, Fang Zheng, Chuanguang Wang, Leiming Ding

**Affiliations:** Department of Anesthesiology, Lishui Municipal Central Hospital, Lishui, Zhejiang 323000, China

## Abstract

**Objective:**

To investigate the effects of ultrasound-guided fascia iliac compartment block (FICB) on patients' postoperative pain and inflammatory factors as well as nucleotide-binding domain and leucine-rich repeat (NLR) family, pyrin domain-containing 3 (NLRP3) in femoral intertrochanteric fracture.

**Methods:**

This single-blind randomized controlled study included 231 patients with femoral intertrochanteric fracture treated in our hospital from January 2017 to December 2020. All patients were randomized into two groups, the FICB group (*n* = 116) and the general anesthesia group (control group, *n* = 115). The serum NLRP3 levels and inflammatory factors were evaluated. The heart rate (HR), mean arterial pressure (MAP), and SpO_2_ values were recorded. Pain condition was measured by the visual analogue scale (VAS) score. Harris score was performed for positive hip function.

**Results:**

The values of HR and MAP were significantly lower after anesthesia induction in FICB groups compared with the control group. However, no significant difference was found for SpO_2_. Compared with the control group, the VAS scores within 72 h after surgery were all markedly lower in the FICB group than in the control group and showed no significant difference at 1 week after surgery. The levels of NLRP3 and interleukin 6 (IL-6) were significantly lower in FICB patients at 1 h, 6 h, 24 h, 48 h, and 72 h after surgery compared with the control group. Tumor necrosis factor-*α* (TNF-*α*) showed a significant lower level in the FICB group at 1 h and 6 h after surgery, and significant lower levels of C-reactive protein (CRP) were found at 1 h and 24 h after surgery compared with the control group. Positive correlation was found between NLRP3 and IL-6, as well as CRP and VAS scores after 1 h of the surgery. No significant difference was found for both Harris score and postoperative complications between the two groups.

**Conclusion:**

Fascia iliac compartment block could reduce the postoperative pain, which might be associated with the decrease of the serum levels of NLRP3, CRP, IL-6, and TNF-*α* in femoral intertrochanteric fracture patients.

## 1. Introduction

The incidence rate of hip fractures is increasing every year, which affects about 18% of the world's women and 6% of the men, especially in the elderly [1–3]. In hip fracture, femoral intertrochanteric fracture is a common fracture in elderly, accounting for about 50% of hip fractures and leading to 15%~20% death after fracture [4, 5]. At present, surgery is still the main treatment strategy for femoral intertrochanteric fracture, including InterTAN intramedullary nail, proximal femoral nail anti-rotation (PFNA), and Asian proximal femoral nail (APFN) [6–8]. Pain is one of the postoperative complications which may influence patients' recovery and treatment experience [9]. Thus, the pain management is of great significance.

Nowadays, many methods are reported to relieve patients' postoperative pain, including use of analgesics and nonsteroidal anti-inflammatory drugs [10, 11]. Among these pain management methods, the application of fascia iliac compartment block (FICB) has been already reported in several surgical types such as total hip arthroplasty (THA) [12, 13]. However, few studies focused on application of FICB in treatment of femoral intertrochanteric fracture alone. Besides, during the pain process, the activation of inflammation-related factors is closely related to pain development [14]. However, the influence of FICB on inflammatory factors is also rarely studied.

In the present study, a randomized control research was performed to investigate the effects of FICB on patients' postoperative pain and inflammatory factors as well as inflammation-related factor NLR family, pyrin domain-containing 3 (NLRP3) in femoral intertrochanteric fracture. This study might provide new clinical evidence for FICB in femoral intertrochanteric fracture.

## 2. Methods and Materials

### 2.1. Patients and Grouping

The present single-blinded randomized control study included a total of 231 cases of femoral intertrochanteric fracture patients who were admitted in our hospital during January 2017 to December 2020. The inclusion criteria were as follows: (1) patients were diagnosed with femoral intertrochanteric fracture by imaging evidence such as X-ray, CT scan, and MRI; (2) patients with American Society of Anesthesiologists (ASA) grades I~III. The following patients were excluded: (1) patients with severe renal, liver, or heart diseases and (2) patients with inflammation or tumors at block position; (3) patients with dysfunction of coagulation; (4) parents who could not cooperate with the measurement of visual analogue scale (VAS) or Harris scale; (5) patients with open fractures; and (6) patients who failed with FICB or quit the study. All patients were randomized into two groups, the FICB group (*n* = 116) and the general anesthesia group (control group, *n* = 115) using a random number table generated by SPSS 18.0 software (SPSS Inc., Chicago, USA). Written informed consent was obtained from all patients. The present study was approved by the ethical committee of Lishui Municipal Central Hospital.

### 2.2. Anesthetic Strategy

All patients received routine preparation before anesthesia, including brief education, helping relieving tension, and fasting and water prohibition for 8 h. Patients all received scopolamine 0.5 mg and diazepam 5 mg before 30 min of the surgery.

For both groups, patients received induced anesthesia under the monitor of a PHILIPS IntelliVue MP60 Monitor (PHILIPS Inc.) by intravenous injection of midazolam (0.05 mg/kg), sufentanil (0.5 *μ*g/kg), propofol (0.5 ~ 2 mg/kg), and rocuronium (0.6 mg/kg). The anesthesia maintenance was performed by intravenous injection of propofol (0.05~0.15 mg/kg/min) and remifentanil (0.15 *μ*g/kg/min). Injection of cisatracurium (0.1 mg/kg) was performed every 30 min during the surgery. The BIS value was maintained within 40~60.

For the FICB group, patients received ultrasound-guided FICB before the above general anesthesia surgery. Briefly, the ultrasonic probe was used to find the femoral artery. An incision was made at 1~2 cm below the position of the outer 1/3 junction of the line between anterior superior iliac spine and pubic symphysis. The nerve stimulation needle was put through fascia lata and iliac fascia to the inferior iliac fascia space under the monitor of an M-Turbo Portable Color Ultrasonic Diagnostic Instrument (SONOSITE Inc.). After injection of 2 ml normal saline, 0.2% ropivacaine (30~40 ml) was injected to the compartment to conduct FICB. The success of FICB was confirmed by acupuncture method. After successful FICB, patients received the above general anesthesia,

The control group only received general anesthesia without FICB.

All patients received internal fixation surgeries including InterTAN intramedullary nail and proximal femoral nail anti-rotation (PFNA). The surgical strategies were made according to the patients' conditions and will. All surgeries were conducted by the same team according to the same protocol.

For both groups, patients received patient-controlled intravenous analgesia pump (PCIA) after surgery containing fentanyl 0.5 *μ*g/kg every time with no background infusion, block time 8 min and limited to 2 *μ*g/kg/h.

All patients receive the routine postoperative treatment including anti-infection (oral antibiotics), antithrombus (low molecular weight heparin), and routine nursing treatment.

### 2.3. Measurement of NLRP3 and Inflammatory Factors

For all patients, venous blood samples (5 ml) were collected at the following time points: before the surgery, 1 h, 6 h, 24 h, 48 h, 72 h, and 1 week after surgery. The serum NLRP3 levels and inflammatory factors of IL-6 and TNF-*α* were evaluated using enzyme-linked immunosorbent assay (ELISA) by corresponding kits purchased from MyBioSource Inc. (NLRP3, cat. No. MBS3802246) and BOSTER Inc. (IL-6 cat. No. EK0410, TNF-*α* cat. No. EK0525). The levels of CRP were measured by using a Hitachi 7600 Automatic Biochemical Analyzer (Hitachi Corporation).

### 2.4. Measurement of Clinical Outcomes and Follow-Up

The clinical characteristics and demographic data of all patients were recorded, including age, sex, preoperative complications, surgical methods, ASA grade, and fracture AO types. The heart rate (HR), mean arterial pressure (MAP), and SpO_2_ values before the surgery (*T*_0_), after induced anesthesia (*T*_1_), and 5 min after surgery (*T*_2_) were recorded. The VAS score was evaluated before the surgery as well as at 1 h, 6 h, 24 h, 48 h, 72 h, and 1 week after surgery. Harris score was performed before surgery and at 3 months after surgery. Complications during admission were also collected. All patients were followed up for 3 months.

### 2.5. Statistical Analysis

Data were expressed by mean ± SD if normally distributed and or median (range) if nonnormally distributed. The rates were analyzed by the chi-square test. The Student *t*-test and Mann–Whitney *U* test were used for analysis of normally and nonnormally distributed data, respectively. Spearman's analysis was conducted for correlation analysis. *P* < 0.05 was considered as statistically different. All calculations were made using SPSS 18.0 (SPSS Inc., Chicago, USA).

## 3. Results

### 3.1. Basic Clinical Characteristics of All Patients

As shown in Table 1, among the 231 patients, 138 patients (59.74%) were with ASA II and 93 patients (40.26%) were with ASA III. The cases of different AO types were 105 cases (45.45%) for *A*_1_, 72 cases (31.17%) for *A*_2_, and 54 cases (23.38%) for *A*_3_. A total of 134 cases (58.01%) received InterTAN intramedullary nail treatment, and 97 cases (41.99%) received PFNA treatment. No significant difference was found for all indices between the two groups.

### 3.2. Intraoperative HR, MAP, and SpO_2_ of the Two Groups

The values of HR, MAP, and SpO_2_ were measured under different time points. It was found that in both groups, HR and MAP values decreased at *T*_1_ and increased at *T*_2_. The values of HR and MAP were significant lower at *T*_1_ in FICB groups compared with the control group (*P* < 0.05, Table 2). However, no significant difference was found for SpO_2_ between the two groups. At *T*_2_ time, no significant difference was found for all indices.

### 3.3. Alteration of VAS Score after Surgery of the Two Groups

The pain condition of the patients was then evaluated. As shown in Figure 1, for all patients, the VAS scores gradually decreased after surgery. Compared with the control group, the VAS scores within 72 h after surgery were all markedly lower in the FICB group than in the control group (*P* < 0.05). However, at 1 week after surgery, the VAS score showed no significant difference.

### 3.4. Dynamic Changes and Correlation of NLRP3 and Inflammatory Factors of the Two Groups

The change of the serum values of NLRP3 and inflammatory factors is shown in Figure 2. It was observed that at 1 h to 24 h after surgery, the levels of NLRP3, CRP, IL-6, and TNF-*α* were all significantly increased compared to their baseline and then gradually decreased. The levels of NLRP3 and IL-6 were significantly lower in FICB patients at 1 h, 6 h, 24 h, 48 h, and 72 h after surgery compared with the control group (*P* < 0.05). TNF-*α* showed significant lower level in the FICB group at 1 h and 6 h after surgery, and significant lower levels of CRP were found at 1 h and 24 h after surgery compared with the control group (*P* < 0.05). No significant difference was found after 1 week of the surgery. Besides, significant positive correlation was found between NLRP3 and IL-6 after 1 h of the surgery (*P* < 0.05, Table 3). Meanwhile, positive correlation was only found between CRP and VAS scores after 1 h of the surgery (*P* < 0.05, Table 4). Other inflammatory factors of CRP, IL-6, and TNF-*α* showed no significant correlation with VAS score.

### 3.5. Harris Score and Postoperative Complications

Finally, the patients' hip function was evaluated. As shown in Table 5, no significant difference was found for Harris score before the surgery between the two groups. At 3 months after surgery, both groups showed markedly increased Harris score than their baseline. However, no significant difference was found for both Harris score and postoperative complications between the two groups.

## 4. Discussion

Femoral intertrochanteric fracture is a common orthopedic disease especially in elderly patients. Although many treatments and surgical methods were developed, the postoperative recovery and pain management keep being a clinical problem. In the present study, we demonstrated that fascia iliac compartment block could reduce the postoperative pain and decrease the serum levels of NLRP3, CRP, IL-6, and TNF-*α* in femoral intertrochanteric fracture patients, with no severe side effects.

Fascia iliac compartment block has been reported in a series of surgeries. It was found that FICB could reduce the postoperative pain of femoral neck fractures compared with the standard analgesia alone [15]. Desmet et al. demonstrated that FICB reduced the morphine consumption after THA [16]. Another study also found that use of FICB might also benefit the postoperative cognitive status; however, the trend was not significant [17]. However, despite these researches, we noticed that no study focused on FICB in treatment of femoral intertrochanteric fractures alone. In the present study, we found that FICB could also reduce the postoperative pain after femoral intertrochanteric fracture. However, FICB did not influence the recovery of hip function.

The change of inflammation is closely related to pain condition. It was found after THA, proinflammatory factors of CRP and IL-6 all increased, which started to decrease after 3 d of the surgery, and local infiltration analgesia could reduce the release of the cytokines [18]. Another study found that synovial fluid PGE2, IL-6, IL-8, and TNF-*α* were all increased after THA and were correlated with numerical rating scale at walking (NRSW) [19]. In a meta-analysis, authors also found that postoperative CRP and IL-6 levels were higher in patients with postoperative cognitive dysfunction after THA [20]. Among these inflammation-related factors, NLRP3 is a newly found factor which is reported to be associated with process of many diseases, including bone injury. It was reported that inhibition of NLRP3 could improve the diabetic-induced impaired fracture healing [21]. NLRP3 was also found to facilitate the release of inflammatory factors in metabolic bone disease and suppress the expression of angiogenesis-related genes during bone formation [22]. However, up to now, few studies reported changes of inflammatory factors and NLRP3 after surgery of femoral intertrochanteric fractures, and the influence of FICB on this change is also unclear. In our research, we observed that both NLRP3 and inflammatory factors of CRP, IL-6, and TNF-*α* were reduced by treatment of FICB. Besides, NLRP3 and inflammatory factors were correlated with VAS score, suggesting that they were associated with postoperative pain condition.

The present study also has some limitations, both small sample size and unclear mechanism for how FICB reduce postoperative pain limited the significance of this study. All these need further researches to improve.

## 5. Conclusion

In summary, through a randomized controlled study, we found that FICB can improve postoperative pain management and the release of NLRP3 and inflammatory factors in femoral intertrochanteric fractures. This study may provide new clinical evidence and research objectives for the application of FICB in femoral intertrochanteric fracture.

## Figures and Tables

**Figure 1:** VAS scores before the surgery as well as at 1 h, 6 h, 24 h, 48 h, 72 h, and 1 week after surgery. ^∗∗∗^*P* < 0.001.

**Figure 2:** Dynamic changes of NLRP3 and inflammatory factors of the two groups. ^∗∗^*P* < 0.01; ^∗∗∗^*P* < 0.001.

**Table 1:** Basic clinical characteristics of all patients.

Characteristics	FICB, *n* = 116	Control, *n* = 115	*P* value^∗^
Age (y)	71.87 ± 6.71	71.47 ± 7.20	0.669
Sex, male (%)	65 (56.03)	60 (52.17)	0.584
ASA grade, *n* (%)			0.671
II	71 (61.21)	67 (58.26)	
III	45 (38.79)	48 (41.74)	
AO types, *n* (%)			0.684
*A*_1_	54 (46.55)	51 (44.35)	
*A*_2_	33 (28.45)	39 (33.91)	
*A*_3_	29 (25.00)	25 (21.74)	
Surgery, *n* (%)			0.287
InterTAN	63 (54.31)	71 (61.74)	
PFNA	53 (45.69)	44 (38.26)	
Complication, *n* (%)			0.766
Diabetes	32 (27.59)	27 (23.48)	
Hypertension	36 (31.03)	34 (29.57)	

^∗^The rates were analyzed by the chi-square test. Student's *t*-test was used for analysis of normally and nonnormally distributed data.

**Table 2:** Intraoperative HR, MAP, and SpO_2_ of the two groups.

Characteristics	Time point	FICB, *n* = 116	Control, *n* = 115	*P* value
HR	*T*_0_	84.31 ± 10.92	82.50 ± 11.23	0.217
	*T*_1_	72.63 ± 11.75	78.03 ± 10.86	<0.001^∗^
	*T*_2_	79.66 ± 10.66	80.12 ± 12.20	0.762

MAP	*T*_0_	86.56 ± 9.02	86.98 ± 9.60	0.736
	*T*_1_	73.96 ± 11.18	78.16 ± 11.50	0.005^∗^
	*T*_2_	80.18 ± 11.91	83.10 ± 10.70	0.051

SpO_2_	*T*_0_	96.88 ± 0.56	96.82 ± 0.59	0.422
	*T*_1_	96.91 ± 0.59	96.88 ± 0.59	0.729
	*T*_2_	96.83 ± 0.54	96.83 ± 0.57	0.952

^∗^ *P* < 0.05.

**Table 3:** Correlation among NLRP3, CRP, IL-6, and TNF-*α* at 1 h after surgery in all patients.

	NLRP3	CRP	IL-6	TNF-*α*
NLRP3				
Person's correlation	—	0.064	0.190	0.034^∗^
*P*	—	0.332	0.004^∗^	0.611
CRP				
Person's correlation	0.064	—	0.009	0.093
*P*	0.332	—	0.897	0.158
IL-6				
Person's correlation	0.190	0.009	—	0.029
*P*	0.004^∗^	0.897	—	0.659
TNF-*α*				
Person's correlation	0.034	0.093	0.029	—
*P*	0.611	0.158	0.659	—

^∗^ *P* < 0.05.

**Table 4:** Correlation among inflammatory factors of NLRP3, CRP, IL-6, and TNF-*α* and VAS score at 1 h after surgery in all patients.

Factors	Person's correlation	*P*
NLRP3	0.044	0.509
CRP	0.184	0.005^∗^
IL-6	0.087	0.187
TNF-*α*	0.079	0.230

^∗^ *P* < 0.05.

**Table 5:** Harris score and postoperative complications.

	FICB, *n* = 116	Control, *n* = 115	*P* value
Harris before	28.44 ± 5.70	28.20 ± 5.45	0.742
Harris at 3 mon	77.53 ± 10.43	77.07 ± 11.70	0.755
Complications, *n* (%)			0.836
Nausea and vomiting	13 (11.21)	15 (13.04)	
Infection	7 (6.03)	9 (7.83)	
Venous thromboembolism	3 (2.59)	2 (1.74)	

## Data Availability

The datasets during the current study are available from the corresponding author on reasonable request.
